# miR-101 targeting ZFX suppresses tumor proliferation and metastasis by regulating the MAPK/Erk and Smad pathways in gallbladder carcinoma

This article has been retracted.

**DOI:** 10.18632/oncotarget.7970

**Published:** 2016-03-08

**Authors:** Run-Fa Bao, Yi-Jun Shu, Yun-Ping Hu, Xu-An Wang, Fei Zhang, Hai-Bin Liang, Yuan-Yuan Ye, Huai-Feng Li, Shan-Shan Xiang, Hao Weng, Yang Cao, Xiang-Song Wu, Mao-Lan Li, Wen-guang Wu, Yi-Jian Zhang, Lin Jiang, Qian Dong, Ying-Bin Liu

**Affiliations:** ^1^ Department and laboratory of General Surgery, Xinhua Hospital, Affiliated with Shanghai Jiao Tong University, School of Medicine, No. 1665 Kongjiang Road, Shanghai 200092, China; ^2^ Institute of Biliary Tract Disease, Shanghai Jiao Tong University School of Medicine, No. 1665 Kongjiang Road, Shanghai 200092, China

**Keywords:** miR-101, ZFX, EMT, TGF-β, gallbladder carcinoma

## Abstract

Gallbladder cancer (GBC), the most common malignancy of the bile duct, is highly aggressive and has an extremely poor prognosis, which is a result of early metastasis. As it is regulated being at multiple levels, the metastatic cascade in GBC is complex. Recent evidence suggests that microRNAs (miRNAs) are involved in cancer metastasis and are promising therapeutic targets. In this study, miR-101 was significantly downregulated in tumor tissues, particularly in metastatic tissues. In GBC patients, low miR-101 expression was correlated with tumor size, tumor invasion, lymph node metastasis, TNM stage, and poor survival. Moreover, miR-101 was an independent prognostic marker for GBC. Additionally, miR-101 inhibited GBC cell proliferation, migration, invasion, and TGF-β-induced epithelial-mesenchymal transition (EMT) *in vitro* and *in vivo*. Mechanistically, the gene encoding the zinc finger protein X-linked (ZFX) was identified as a direct target of miR-101. More importantly, miR-101 significantly reduced activation of the MAPK/Erk and Smad signaling pathways, resulting in inhibition of TGF-β-mediated induction of EMT. Altogether, our findings demonstrate a novel mechanism by which miR-101 attenuates the EMT and metastasis in GBC cells and suggest that miR-101 can serve as a potential biomarker and therapeutic target for GBC management.

## INTRODUCTION

Gallbladder carcinoma (GBC), the most common malignancy of the bile duct, is a highly aggressive neoplasm associated with high mortality and an extremely poor prognosis [1, 2]. Despite recent diagnostic and therapeutic advances, the 5-year survival rate for GBC is only 13–30% [3]. Because of the absence of specific symptoms and signs, GBC is usually detected at an advanced stage [4]. To date, surgical resection is the only potentially curative therapy for GBC [5]; however, even after complete resection, loco-regional recurrence rates are extremely high [6] due to early metastasis via lymphatic, perineural, and hematogenous routes, as well as direct invasion into the liver [7]. All other treatments, including chemotherapy and radiotherapy, are palliative and do not markedly improve prognosis and survival [8]. Therefore, the identification of novel and effective therapeutic targets for GBC is urgently required.

MicroRNAs (miRNAs) are highly conserved non-coding regulatory RNAs of 17 to 25 nucleotides in length [9]. As post-transcriptional regulators, miRNAs can negatively regulate gene expression by binding directly to the 3′ untranslated regions (3′UTRs) of corresponding target messenger RNAs (mRNAs) in a sequence-specific manner, thereby inducing mRNA degradation or protein translation repression [10]. miRNAs act as either tumor suppressors or carcinogenic agents in several cancers [11]. For example, miR-101 has been established as a tumor suppressor with inhibitory effects on cell proliferation, migration, and invasion. In particular, low miR-101 levels have been found in gastric cancer, non-small cell lung cancer, colorectal cancer, and hepatocellular carcinoma [12–15]; however, it remains unclear whether miR-101 is involved in the progression and metastasis of GBC.

In the present study, we first elucidated the function of miR-101 in GBC by analyzing miR-101 expression in human GBC samples and cell lines and by investigating the effects of ectopically expressed miR-101 on GBC cell proliferation and metastasis. Additionally, we demonstrated that attenuation of the epithelial-mesenchymal transition (EMT) and inhibition of the MAPK/Erk and Smad signaling pathways may promote the tumor-suppressive role of miR-101 in GBC. Furthermore, we identified that the gene encoding the zinc finger protein X-linked (ZFX) is a direct target of miR-101, suggesting that the TGF-β/miR-101/ZFX axis plays an important role in GBC progression and may therefore serve as a potential therapeutic target for GBC.

## RESULTS

### Downregulation of miR-101 is associated with poor prognosis in GBC patients

In analyzing primary tumor specimens from 53 patients with GBC by qRT-PCR, miR-101 expression was found to be significantly lower in tumor tissues than corresponding non-tumor tissues (Figure 1A and 1B). We compared low (27 cases) and high (26 cases) miR-101 expression groups (Table 1) and found that low miR-101 expression was significantly correlated with tumor size (*P*=0.027), tumor invasion (*P*=0.005), lymph node metastasis (*P*=0.028), and TNM stage (*P*=0.002). Furthermore, miR-101 expression was significantly lower in the 25 cases with clinicopathologically confirmed metastasis compared to the 28 cases without metastasis (*P*<0.05) (Figure 1C). Kaplan-Meier analysis revealed that low miR-101 expression was associated with shorter overall survival (*P*<0.01) (Figure 1D). The mean survival in the low miR-101 expression group was 8.7 months, while in the high miR-101 expression group was 20.2 months. Multivariate Cox regression analysis showed low miR-101 expression (*P*<0.001) and TNM stage to be independent prognostic factors of patient survival (Table 2).

**Figure 1:** miR-101 expression is downregulated in GBC **A.** miR-101 expression in GBC tissues and corresponding non-tumor tissues as measured by qRT-PCR (**P<0.01). **B.** Relative miR-101 expression levels in 53 GBC patients. **C.** Relative miR-101 expression levels in primary tumor samples with or without clinicopathologically confirmed metastasis (*P<0.05). **D.** Kaplan-Meier analysis of the correlation between miR-101 expression and overall survival in GBC patients. Patients with low miR-101 expression had significantly shorter overall survival (*P*<0.01).

**Table 1:** Association of miR-101 expression with the clinicopathological characteristics of GBC

Characteristics	Cases	miR-101 expressiom (%)		χ^2^ value	*P* value
		Low	High		
Sex					
*Male*	18	7 (38.9%)	11 (61.1%)	1.585	0.254
*Female*	35	20 (57.1%)	15 (42.9%)		
Age (yr)					
*<60*	13	7 (53.8%)	6 (46.2%)	0.058	1.000
*≥60*	40	20 (50.0%)	20 (50.0%)		
Gallbladder stone					
*Present*	36	19 (52.8%)	17 (47.2%)	0.151	0.773
*Absent*	17	8 (47.1%)	9 (52.9%)		
Tumor size					
*<4 cm*	30	11 (36.7%)	19 (63.3%)	**5.638**	0.027*
*≥4 cm*	23	16 (69.6%)	7 (30.4%)		
Histology differentiation					
*Well*	5	1 (20.0%)	4 (80.0%)	3.010	0.222
*Moderate*	21	13 (61.9%)	8 (38.1%)		
*Poor*	27	13 (48.1%)	14 (51.9%)		
Tumor invasion (AJCC)					
*Tis.-T2*	22	6 (37.2%)	16 (62.8%)	**8.433**	0.005*
*T3-T4*	31	21 (58.8%)	10 (41.2%)		
Lymph node metastasis					
*Present*	28	10 (27.3%)	18 (72.7%)	**5.509**	0.028*
*Absent*	25	17 (68.0%)	8 (32.0%)		
TNM stage (AJCC)					
*0-II*	19	4 (21.1%)	15 (78.9%)	**10.589**	0.002*
*III-IV*	34	23 (67.6%)	11 (32.4%)		

* Statistically significant difference; AJCC, American Joint Committee on Cancer.

**Table 2:** Univariate and multivariate analysis of the association of prognosis with clinicopathological characteristics and miR-101 expression in GBC patients

Characteristics	Univariable analysis		Multivariable analysis	
	HR (95% CI)	*P* value	HR (95% CI)	*P* value
Sex *(male vs. female)*	0.926 (0.465~1.845)	0.826		
Age *(<60 vs. ≥60)*	1.007 (0.466~2.179)	0.985		
Gallbladder stone	0.830 (0.412~1.672)	0.598		
*(present vs. absent)*				
Tumor size	1.281 (0.650~2.521)	0.470		
*(< 4 cm vs. ≥ 4 cm)*				
Histology differentiation	0.745 (0.434~1.280)	0.480		
*(well or moderate vs. poor)*				
Tumor invasion (AJCC)	**2.728 (1.292~5.760)**	0.006*	0.808 (0.184~3.558)	0.778
*(Tis.-T2 vs. T3-T4)*				
Lymph node metastatis	**2.463 (1.230~4.934)**	0.008*	1.138 (0.477~2.716)	0.771
*(present vs. absent)*				
TNM stage (AJCC)	**3.408 (1.519~7.643)**	0.002*	**2.431 (1.010~5.847)**	0.047*
*(0-II vs. III-IV)*				
MiR-101 expression	**0.296 (0.144~0.606)**	<0.001*	**0.406 (0.186~0.883)**	0.023*
*(low vs. high)*				

* Statistically significant difference; AJCC, American Joint Committee on Cancer; CI, confidence interval; HR, hazard ratio.

### miR-101 inhibits GBC cell proliferation *in vitro*

To investigate the biological functions of miR-101 in GBC development, miR-101 expression was measured in five GBC cell lines (Figure 2A). The GBC-SD and NOZ cell lines, which possess the highest potential of metastasis among the cell lines tested, had the lowest miR-101 expression. To functionally characterize miR-101 in GBC, we restored miR-101 levels by ectopically expressing the miRNA in GBC-SD and NOZ cells. According to qRT-PCR results, higher miR-101 expression was achieved after transfection with miR-101 mimics compared to miR-NC (Figure 2B). CCK-8 and colony formation assays were performed to assess the role of miR-101 in GBC-SD and NOZ cell proliferation. The GBC cells transfected with miR-101 clearly grew slower than the control group (Figure 2C). Moreover, the number and the mean size of the colonies formed by the GBC-SD and NOZ cells were significantly decreased following transfection with miR-101 (Figure 2D and Supplementary Figure S1), which is consistent with miR-101 exerting an inhibitory function in GBC cell proliferation.

**Figure 2:** Functional analysis of miR-101 *in vitro* **A.** miR-101 expression in 5 human GBC cell lines. **B.** miR-101 expression following transfection of GBC-SD and NOZ cells as confirmed by qRT-PCR (**P<0.01). **C.** Cell growth rates after miR-101 transfection as determined by CCK-8 proliferation assays conducted at various time points (**P<0.01). **D.** Representative images of colony formation induced by miR-101 in GBC cells. The mean number of colonies is shown in the right panel (**P<0.01). **E.** GBC cells transfected with miR-101 were stained with annexin V-FITC/PI and analyzed by flow cytometry. The percentage of apoptotic cells is presented in the bottom panel (**P<0.01). **F.** The cell cycle phases of the treated cells were evaluated by flow cytometry. The percentage of each phase is presented in the bottom panel (**P<0.01).

### miR-101 promotes GBC cell apoptosis and induces cell cycle disorder

To explore the molecular mechanism by which miR-101 regulates GBC cell proliferation, the effects of miR-101 on apoptosis and the cell cycle were investigated by flow cytometry. The apoptotic rate was significantly increased in miR-101-transfected cells compared to control cells (41.97 vs. 11.86% of GBC-SD cells and 16.97 vs. 3.04% of NOZ cells, *P*<0.01) (Figure 2E). Cell cycle analysis of GBC-SD and NOZ cells revealed fewer in G0/G1 phase and more in S and G2/M phases compared to the control group (Figure 2F). These data indicate that exogenous miR-101 induced GBC cell apoptosis and cell cycle disorder.

### miR-101 inhibits GBC cell migration and invasion

To investigate the effects of miR-101 on cancer cell migration and invasion, we performed wound healing and transwell assays *in vitro*. Transwell assays with or without Matrigel demonstrated that GBC-SD and NOZ cells transfected with miR-101 had lower invasive activity than control cells (*P*<0.01; Figure 3A). The wound healing assay showed that increased miR-101 expression in GBC-SD and NOZ cells was associated with significantly slower wound closure (*P*<0.01, Figure 3B). Migration in GBC-SD and NOZ cells transfected with miR-101 was inhibited by EMT-like changes, as shown by increased expression of the epithelial markers E-cadherin and β-catenin and decreased expression of the mesenchymal marker vimentin (Figure 3C). These results indicate that miR-101 inhibits GBC cell proliferation and metastasis *in vitro*.

**Figure 3:** miR-101 inhibits GBC cell migration and invasion **A.** Migration (upper panel) and invasion (bottom panel) assays were conducted using GBC cells transfected with miR-101. Quantitative results are shown in the right panel (**P<0.01). **B.** Wound healing assays were used to detect GBC cell motility following transfection with miR-101. Wound closure percentages are shown in the right panel (**P<0.01). **C.** Expression of EMT biomarker proteins in GBC cells with and without miR-101 transfection was examined by immunofluorescence analysis. The green signals represent staining for E-cadherin, whereas the red signals represent staining for β-catenin or vimentin. Nuclei were counterstained with DAPI.

### miR-101 inhibits GBC cell proliferation and metastasis *in vivo*

After incubation with miR-101 mimics or miR-NC, approximately 2.5×10^6^ NOZ cells were injected into the right flank subcutaneous tissues of nude mice. Three weeks after inoculation, the mice were euthanized, and the xenografted tumors were excised. As shown in Figure 4A, tumor growth was significantly inhibited in the presence of miR-101 (*P*<0.01). IHC staining confirmed that E-cadherin, β-catenin, and vimentin expression produced similar trends to those found in the above-described *in vitro* experiments (Figure 4C). Next, we employed a liver tumor metastasis model created via splenic injection to monitor NOZ cell metastasis *in vivo*. Compared to the miR-101-treated mice, the total metastasis number was markedly higher in the control mice (Figure 4B). Collectively, our data demonstrate that miR-101 plays a potential role in promoting cell proliferation and metastasis both *in vitro* and *in vivo*.

**Figure 4:** miR-101 suppresses GBC cell proliferation and metastasis *in vivo* **A.** Mice bearing subcutaneous xenografts of NOZ cells were euthanized after 3 weeks of treatment with miR-101. The right panels show tumor volume and weight (**P<0.01). **B.** A liver metastasis tumor model was created via splenic injection to evaluate the anti-metastatic role of miR-101. The total metastasis in each group is shown by the histogram in the right panel (**P<0.01). **C.** Paraffin sections were stained for IHC with antibodies against E-cadherin, β-catenin, and vimentin.

### ZFX is a direct downstream target of miR-101

To explore the molecular mechanisms by which miR-101 regulates GBC cell proliferation and metastasis, the miRDB (www.mirdb.org) and TargetScan (www.targetscan.org) databases were used to predict targets of miR-101. ZFX was identified as a potential target, and we performed a luciferase reporter assay to determine whether ZFX is indeed regulated by miR-101. To accomplish this, we constructed 3′UTR reporter plasmids encoding full-length wild type or mutant miR-101 binding sites for ZFX (Figure 5A). We found that miR-101 repressed the reporter activity of the wt-ZFX-3′UTR plasmid but not that of the mut-ZFX-3′UTR plasmid (Figure 5B). qRT-PCR and western blot analysis confirmed that miR-101 suppressed the endogenous expression of ZFX at the protein level but not at the mRNA level (Figure 5C and 5D). These results indicate that ZFX is a direct downstream target of miR-101.

**Figure 5:** ZFX is a direct downstream target of miR-101 **A.** Putative miR-101-binding sequence within the 3′UTR of ZFX mRNA. Mutations in the complementary site for the seed region of miR-101 in the 3′UTR of the ZFX gene are indicated. **B.** Reporter plasmids containing either the wild type 3′UTR or a mutated 3′UTR of the ZFX gene were co-transfected into 293T cells with an miR-101-encoding plasmid, and luciferase activity was measured. The data are presented as the mean ± SD of three experiments. **C.** ZFX mRNA expression after miR-101 transfection was detected by qRT-PCR. **D.** ZFX expression in miR-NC- and miR-101-transfected GBC cells was analyzed by western blot analysis. β-actin was used as a loading control. GBC cells were transfected with an miR-NC/empty vector, an miR-101/empty vector, or an miR-101/ZFX plasmid. **E.** Cell growth rates were determined using a CCK-8 proliferation assay (**P<0.01). **F.** Transwell migration and invasion assays were performed, and the results are shown in the right panel (**P<0.01). **G.** Wound healing assays were used to detect cell motility after transfection. The wound closure percentages are shown in the right panel (**P<0.01).

### ZFX overexpression rescues the effects of miR-101 on GBC cell proliferation and metastasis

Rescue experiments were performed to further assess whether the effects of miR-101 on GBC cell proliferation and metastasis are indeed mediated by ZFX. GBC-SD and NOZ cells were transfected with either a ZFX overexpression plasmid or an empty vector, and transfection efficiencies were detected by fluorescence microscopy and qRT-PCR. The results indicated that the transfections were effective (Supplementary Figure S2A and S2B). Using a CCK-8 assay, we found that ZFX overexpression partially reversed the miR-101-dependent inhibition of GBC cell proliferation (Figure 5E). Moreover, restoration of ZFX expression significantly attenuated the miR-101-mediated inhibition of GBC cell migration and invasion (Figure 5F and 5G). IHC confirmed that ZFX expression was significantly higher in human and mouse tissues with low miR-101 expression compared to those with high miR-101 expression (Figure 6A).

**Figure 6:** miR-101 targeting ZFX attenuates MAPK/Erk and Smad signaling **A.** ZFX expression was detected by IHC in human and mouse tumor tissues. **B.** E-cadherin, β-catenin, vimentin, p-Smad2, p-c-Raf, MEK1/2, p-MEK1/2, Erk1/2, and p-Erk1/2 expression was analyzed by western blot analysis in cells transfected with an miR-NC/empty vector, an miR-101/empty vector, or an miR-101/ZFX plasmid. β-actin was used as a loading control. **C.** Representative figures and data from transwell assays conducted using GBC cells treated with 10 ng/mL TGF-β for 0, 24, and 48 h. **D.** Western blot analysis of E-cadherin, β-catenin, vimentin, and ZFX expression in GBC cells following treatment with TGF-β for 0, 24, and 48 h. **E.** Relative expression of ZFX mRNA in GBC cells treated with TGF-β for 0, 24, and 48 h.

### miR-101 attenuates MAPK/Erk and smad signaling by targeting ZFX

To explore the molecular mechanism underlying EMT control by miR-101/ZFX, western blot analyses were performed to identify EMT biomarkers and the phosphorylation statuses of proteins involved in EMT signaling. As shown in Figure 6B, GBC cells transfected with miR-101 showed increased expression of E-cadherin and β-catenin and decreased expression of vimentin, indicating that EMT was inhibited in these cells. Moreover, miR-101 significantly reduced the phosphorylation of c-Raf, MEK, Erk1/2, and Smad2 in GBC-SD and NOZ cells. These changes were partially recovered by re-introducing ZFX, indicating that miR-101/ZFX functions as a key mediator of EMT via the MAPK/Erk and Smad signaling pathways.

To further elucidate the relationship between ZFX and TGF-β signaling in GBC, we analyzed the effect of introducing recombinant TGF-β into GBC-SD and NOZ cells. As shown in Figure 6C, time-dependent increases in tumor cell invasive ability were observed after treatment with TGF-β. We also found that TGF-β expression was stimulated as the cells adopted a classical EMT phenotype, which was determined by changes in EMT biomarkers. These changes led to a significant, time-dependent increase in ZFX expression at both the mRNA and protein levels (Figure 6D and 6E).

### miR-101 attenuates EMT in TGF-β-treated GBC cells

To further explore the role of miR-101 in miR-101/ZFX-mediated EMT and GBC cell invasiveness, we transfected miR-101 into GBC-SD and NOZ cells and treated the cells with TGF-β. Transfection of miR-101 partially inhibited the cells from undergoing EMT-like changes. As shown in Figure 7A and 7B, wound-healing and transwell assay results showed that exogenous miR-101 significantly neutralized the effects of TGF-β on cell invasiveness and migration. Moreover, exogenous miR-101 inactivated EMT-associated signaling events that were induced by TGF-β treatment. Western blot analysis showed that miR-101 increased the expression of epithelial markers E-cadherin and β-catenin and suppressed the phosphorylation of c-Raf, MEK, Erk, and Smad2. Simultaneously, miR-101 downregulated the expression of the mesenchymal marker vimentin in cells treated with TGF-β (Figure 7C).

**Figure 7:** miR-101 inhibits EMT in TGF-β-treated GBC cells Representative figures and data from transwell assays **A.** and wound healing assays **B.** conducted using GBC cells transfected with miR-101 and/or TGF-β for 24 h (**P<0.01). **C.** E-cadherin, β-catenin, vimentin, p-Smad2, p-c-Raf, MEK1/2, p-MEK1/2, Erk1/2, and p-Erk1/2 expression was analyzed by western blot analysis in cells transfected with miR-101 and/or TGF-β for 24 h. β-actin was used as a loading control. **D.** A hypothetical model illustrating the role of miR-101 on GBC cells.

## DISCUSSION

Accumulating evidence indicates that miRNAs contribute to cancer pathogenesis. As miRNAs may serve as tumor suppressors or oncogenes, dysregulation of miRNAs is associated with cancer initiation and progression [16]. In the current study, we evaluated miR-101 expression in GBC human tumor tissues and cell lines. We also for the first time explored the biological role and regulatory mechanism of miR-101 in GBC, confirming that miR-101 expression was downregulated in GBC tumor tissues compared to non-tumor tissues. Moreover, miR-101 expression was significantly correlated with adverse clinicopathological factors, such as tumor size, tumor invasion, lymph node metastasis, and TNM stage. We then identified miR-101 as an independent prognostic biomarker for GBC patients by multivariate analysis. In addition, reduced expression of miR-101 was associated with worse overall survival in GBC patients. Collectively, our results demonstrate that miR-101 not only serves as a potential diagnostic biomarker for GBC but also may help predict metastasis or prognosis with high accuracy.

As a tumor-suppressive miRNA species, miR-101 has been reported to suppress cell proliferation and metastatic ability in bladder, liver, breast, and prostate cancer cells [17–19]. In the present study, ectopic expression of miR-101 suppressed GBC cell proliferation, migration, and invasion both *in vitro* and *in vivo*. Furthermore, miR-101 overexpression induced apoptosis and cell cycle disorders in GBC-SD and NOZ cells. This study confirms the tumor-suppressive role of miR-101 in GBC cells and provides evidence for the potential usefulness of miR-101 for miRNA-based cancer therapy.

miR-101 has many predicted targets, including oncogenes, such as stathmin 1 (STMN1), vascular endothelial growth factor C (VEGF-C), and myeloid cell leukemia-1 (Mcl-1) [15, 20, 21]. ZFX is encoded by a gene located on the X chromosome and plays key roles in controlling the self-renewal of embryonic and hematopoietic stem cells [22]. Recently, ZFX was shown to be involved in various physiological functions, including proliferation, differentiation, cell cycle, and cell death [23], and ZFX is highly expressed in malignant tumors, such as renal carcinoma, gastric carcinoma, and colorectal cancer [24–26]. In previous studies, we demonstrated that ZFX expression was significantly correlated with clinical biological behaviors and represented a significant prognostic marker for total post-operative survival in GBC [27, 28]. In the present study, we demonstrated using a luciferase reporter assay that miR-101 could bind to a sequence within the 3′UTR of ZFX. Importantly, ectopic expression of ZFX effectively impeded the ability of miR-101 to inhibit proliferation and metastasis. Our study provides evidence to support the role of miR-101 in inhibiting GBC proliferation and metastasis via the direct targeting of ZFX.

EMT plays a critical role in cancer progression and metastasis. Cancer cells undergoing EMT acquire invasive properties. Numerous studies have illustrated that EMT is a common molecular mechanism in cancer metastasis, and many proteins contribute to this process [29, 30]. Accordingly, we hypothesized that miR-101 is involved in EMT-mediated GBC metastasis. We found that miR-101 expression was closely associated with EMT marker levels. *In vitro* and *in vivo* studies showed that exogenous introduction of miR-101 inhibited GBC cell invasiveness. Our results suggested that miR-101 likely participates in EMT-associated GBC progression. Therefore, this study provides useful insights into the mechanism underlying GBC metastasis.

In addition to the above, we demonstrated that miR-101 inactivates the MAPK/Erk and Smad signaling pathways by affecting protein phosphorylation status, which has been recognized as a pivotal driver of cancer progression. TGF-β induces EMT via both the Smad signaling pathway and complementary pathways, such as the MAPK and PI3K/AKT pathways [31–34]. In the MAPK pathway, Erk activation is a Smad-independent event required for TGF-β-mediated induction of EMT [35, 36]. According to recent studies, abnormal Erk activation plays an important role in diverting the TGF-β-induced EMT in epithelial cells [37]. Previous studies have shown that Erk is rapidly activated by TGF-β in cell culture models of EMT. Furthermore, specific inhibition of MEK inhibits cells from adopting key morphological features associated with EMT [38]. Raf activation confers protection against TGF-β-induced apoptosis by enhancing the proinvasive effects of TGF-β [39]. Similarly, our data indicate that miR-101-induced MAPK/Erk and Smad pathway inactivation occurs via the dephosphorylation of c-Raf, MEK, Erk, and Smad2. Moreover, the inactivation of the two pathways was partially rescued by the re-introduction of ZFX.

Because TGF-β is one of the most potent cytokines linked to inflammation and metastasis in numerous types of cancers [40], we assessed whether miR-101 is involved in pathogenic TGF-β-induced EMT-like changes. We verified that TGF-β promoted GBC cell invasion and migration; we also observed that ZFX expression increased in a time-dependent manner after treatment with TGF-β. Moreover, TGF-β-mediated enhancement of cell migration and invasion was attenuated after incubation with miR-101, which was further verified by western blotting to detect several EMT-related proteins and pathway components. Thus, in GBC, miR-101 appears to be a significant downstream inhibitor of TGF-β signaling, which attenuates the proinvasive effects of TGF-β in GBC cells.

In conclusion, we found that miR-101 expression is downregulated in GBC tissues, particularly in metastatic tissues, and this downregulation is correlated with disease progression. miR-101 potently inhibited GBC cell proliferation and metastasis *in vitro* and *in vivo*, largely mediated by ZFX, a direct target of miR-101. Thus, the miR-101/ZFX axis plays a critical role in TGF-β-mediated induction of EMT via the MAPK/Erk and Smad signaling pathways. Collectively, our results indicate that targeting the miR-101/ZFX axis may serve as a novel diagnostic and therapeutic strategy for managing GBC patients.

## MATERIALS AND METHODS

### Tissue specimens and patient characterization

This study was approved by the Research Ethics Committee of Xinhua Hospital. Informed written consent for the acquisition and storage of medical information was obtained from all patients. Tissue specimens were obtained from 53 GBC patients who underwent radical cholecystectomy at the Department of General Surgery, Xinhua Hospital (Shanghai, China) from January 2011 to December 2014. The samples were either snap-frozen in liquid nitrogen and stored at −80°C for RNA extraction or formalin-fixed and paraffin-embedded for immunohistochemistry (IHC). None of the enrolled patients received pre-operative radiotherapy or chemotherapy. All of the tumors were clinically and histologically diagnosed as GBC. The clinicopathological features of the enrolled patients are shown in Table 1.

### Cell lines and cell culture

The human gallbladder cancer cell lines GBC-SD, SGC-996, NOZ, OCUG, and EHGB-1 were purchased from the Cell Bank of Type Culture Collection of Chinese Academy of Sciences (Shanghai, China). GBC-SD, OCUG, and EHGB-1 cells were cultured in high-glucose DMEM (Gibco, USA). SGC996 cells were cultured in RPMI 1640 medium (Gibco). NOZ cells were cultured in William's medium (Gibco). All of the above media were supplemented with 10% fetal bovine serum (FBS, Gibco), 100 μg/mL streptomycin, and 100 U/mL penicillin (Hyclone, USA). The cells were maintained at 37°C in a humidified atmosphere with 5% CO_2_. For TGF-β treatment, cells were stimulated with 10 ng/mL human recombinant TGF-β1 (Peprotech, USA) diluted with serum-free medium containing BSA for 24 or 48 h.

### RNA extraction and quantitative real-time PCR

Total RNA was extracted from tissue samples or cells with TRIzol reagent (Takara, Shiga, Japan). cDNA was synthesized from 2 μg of total RNA using random primers and MMLV Reverse Transcriptase (Invitrogen, Carlsbad, CA, USA). miRNA and mRNA levels were quantified by quantitative real-time PCR (qRT-PCR) using SYBR® Green (Takara). U6 small nuclear RNA (RNU6B, Life Technologies) and GAPDH served as endogenous controls. The qRT-PCR results were analyzed and shown as relative miRNA or mRNA levels based on cycle threshold (CT) values, which were converted into fold changes. The primer sequences used are listed in Supplementary Table S1.

### RNA oligonucleotides, plasmid construction, and cell transfection

Hsa-miRNA mimics and their cognate control RNAs were purchased from Ribobio (Guangzhou, China). Full-length ZFX cDNA (GenBank accession number NM_001178084.1) was cloned into a GV143 expression vector (Genechem, Shanghai, China). An empty vector was used as a control. Transfection was performed using Lipofectamine 2000 transfection reagent (Invitrogen) according to the manufacturer's instructions. Typically, a 50 nmol/L concentration of miRNA mimics was used for transfection of the RNA oligonucleotides. For plasmid transfections, 3 μg of DNA was used in a 6-well plate, and G418 (200 μg/mL) was added 24 h after transfection. For rescue experiments, 1 μg of plasmid was used in a 6-well plate. The sequences of the miRNAs used are listed in Supplementary Table S1.

### *In vitro* tumorigenesis assays

Cell proliferation was evaluated using a Cell Counting Kit-8 (CCK-8) assay according to the manufacturer's instructions (Dojindo, Kumamoto, Japan). The absorbance values of GBC-SD and NOZ cells at various time points after transfection were measured using a microplate reader (Bio-Rad, Hercules, CA, USA). To perform colony formation assays, 400 cells were seeded per well in 6-well plates and cultured for 14 days. The resulting colonies were fixed with 4% paraformaldehyde and stained with 5% Giemsa (Sigma, St. Louis, MO, USA). The total number of colonies was manually counted. Stained single clones were observed under a microscope (Leica, Germany).

### Annexin V/PI staining assay for apoptosis

At 48 h after transfection, cells were resuspended to a concentration of 1 × 10^6^ cells/mL. Then, 100 μL of binding buffer containing 2.5 μL annexin V-FITC and 1 μL 100 μg/mL PI were added, and the cells were incubated for 30 min in the dark. Following this, the samples were analyzed by flow cytometry (BD, San Diego, CA, USA).

### Cell cycle analysis by flow cytometry

After transfection for 48 h, both floating and adherent cells were collected, washed with cold phosphate-buffered saline (PBS), and fixed with 70% ethanol overnight at 4°C. The cells were then treated with staining buffer (PBS containing 1 mg/mL PI and 10 mg/mL RNase A; Sigma-Aldrich) at 37°C in the dark for 30 min. Following this, the samples were analyzed by flow cytometry (BD).

### *In vitro* migration and invasion assays

Cell migration and invasion assays were performed in a 24-well transwell plate with 8-μm polyethylene terephthalate membrane filters (Costar, Corning, MA, USA). GBC-SD (2×10^4^) and NOZ (3×10^4^) cells in 500 μL of serum-free medium were added to the upper chambers, which contained either uncoated or Matrigel-coated membranes. Each lower chamber was filled with 500 μL medium with 10% FBS. After 24 h of incubation, the filters were removed, and the non-migrating cells on the upper sides of the filters were detached using cotton swabs. The filters were fixed with 4% paraformaldehyde for 15 min. The cells located in the lower filters were stained with Giemsa for 20 min. Migrated or invaded cells were counted in five randomly chosen fields (×100 magnification) per well. For wound healing assay, transfected GBC-SD and NOZ cells were seeded into 6-well plates and grown to confluence. Wounds were created by scraping the confluent cell monolayers with a 200-μL pipette tip. After the cells were extensively rinsed to remove cellular debris, they were cultured in FBS-free media. Photomicrographs were taken under a microscope (Leica) at 0 and 48 h. The percent change in migration was determined by comparing differences in wound width.

### Immunofluorescence analysis

The transfected cells were seeded in 12-well plates and cultured overnight. Then, the cells were fixed in 4% paraformaldehyde and permeabilized in a solution of 0.1% BSA and 0.5% Triton X-100 at room temperature. After washing to remove the blocking solution, the cells were incubated with primary antibodies against β-catenin, E-cadherin, or vimentin for 60 min at 37°C and then washed twice with 0.1% BSA. After 60 min of incubation at 37°C with Cy3 or FITC-conjugated goat anti-rabbit IgG (Beyotime, Shanghai, China), the cells were counterstained with DAPI and imaged under a fluorescence microscope (Leica).

### Luciferase reporter assay

Luciferase assays were performed on 293T cells using the pMIR-REPORT System (Applied Biosystems, USA) following the manufacturer's protocol. Briefly, either the pMIR-REPORT-ZFX-WT-3′UTR plasmid or a mutant form of the plasmid (3 μg) was co-transfected with a pMIR-REPORT β-gal control plasmid (1 μg) into 293T cells (10^6^) with or without miR-101 overexpression using 15 mL of Lipofectamine 2000 (Invitrogen). Twenty-four hours later, luciferase activity was measured using a Luciferase Assay Kit (Applied Biosystems). To accomplish this, lysis solution (250 mL) was added to the cells, and the cells were detached from the plate with a cell scraper. The cell lysate was then transferred into a microfuge tube and centrifuged at 4°C for 5 min. The resulting supernatant was transferred into a fresh tube, and 50 mL of cell extract was transferred into a luminometer tube. Following this, 100 mL of Substrate A (ATP solution) and 100 mL of Substrate B (luciferin solution) were added. Following a 2-s pre-measurement delay, a luminometer was used to measure light emission from the tube for 10 s. β-galactosidase activity was tested using a β-Gal Assay Kit (Invitrogen) following the manufacturer's instructions. Relative luciferase activity was obtained by normalizing luciferase expression against β-gal expression.

### Immunohistochemical analysis

Staining for IHC was performed using a standard immunoperoxidase staining procedure. Sections were incubated overnight at 4°C using primary antibodies against ZFX, E-cadherin, β-catenin, and vimentin. After washing with PBS, the sections were incubated with biotinylated secondary antibodies, followed by further incubation with streptavidin-horseradish peroxidase complex. The sections were then immersed in DAB for 5-10 min and counterstained with 10% Mayer's hematoxylin.

### Western blot analysis

Cells were washed twice with PBS and lysed with RIPA buffer supplemented with protease inhibitors. Protein concentration was measured using a BCA protein assay (Thermo Scientific, Rockford, USA). Proteins were separated using SDS-PAGE electrophoresis and transferred to PVDF membranes. The membranes were blocked and then probed with primary antibodies against ZFX (1:500; Sigma), E-cadherin, β-catenin, vimentin, p-smad2 (1:500; Abcam, MA, USA), p-c-Raf, MEK1/2, p-MEK1/2, ERK1/2, p-ERK1/2, and β-actin (1:1,000; Cell Signaling Technology, Danvers, USA). After incubation with a secondary antibody, immunocomplexes were visualized by enhanced chemiluminescence (Millipore, Billerica, MA). β-actin was used as a loading control.

### Subcutaneous and liver metastasis tumor models in nude mice

Four- to six-week-old BALB/c athymic nude mice were purchased from the Shanghai Laboratory Animal Center of the Chinese Academy of Sciences (Shanghai, China). The mice were housed under specific-pathogen-free conditions following the guidelines of the Ethics Committee of Xinhua Hospital. NOZ cells were treated with miR-101 mimics (200 nM) for 3 days; miR-NC mimics (200 nM) were used as a negative control. To create a subcutaneous xenograft tumor model, 2.5×10^6^ cells (in 100 μL of PBS) were subcutaneously injected into the 2 groups (5 mice/group). One week after tumor cell inoculation, the mice were treated with miR-101 mimics (5 nmol each) or miR-NC mimics (5 nmol each) via multiple-center intratumoral injections twice a week for 2 weeks. Tumor size was measured with a caliper every 3 days for up to 21 days. Tumor growth rates were analyzed by measuring tumor length (L) and width (W) and calculating tumor volume with the formula LW^2^/2. On day 21, the mice were euthanized, and the xenografted tumors were excised, weighed, and examined by IHC. To create a liver tumor metastasis model, NOZ cells were treated with the same mimics described above, and 1.0×10^6^ cells in 200 μL of PBS were injected into the liver via the spleen. After a 5-week incubation, the mice (5 mice/group) were euthanized, and their livers were harvested. The number of metastases was counted.

### Statistical analysis

All experiments were performed in triplicate. The data are expressed as the mean ± SD. miR-101 levels in tumors and paired non-tumor tissues were compared using the paired Student's *t*-test. The independent Student's *t*-test was used to compare the mean values of the two groups. The Pearson χ^2^ test was used to analyze the association of miR-101 expression with clinicopathologic features. Kaplan-Meier plots and log-rank tests were used for survival analysis. Univariate and multivariate Cox proportional hazards regression models were used to analyze independent prognostic factors. *P*<0.05 was considered statistically significant.

## SUPPLEMENTARY FIGURES AND TABLE


